# Differentiating Central Lung Tumors from Atelectasis with Contrast-Enhanced CT-Based Radiomics Features

**DOI:** 10.1155/2021/5522452

**Published:** 2021-11-15

**Authors:** Rui Chai, Qi Wang, Pinle Qin, Jianchao Zeng, Jiwei Ren, Ruiping Zhang, Lin Chu, Xuting Zhang, Yun Guan

**Affiliations:** ^1^School of Data Science, North University of China, 3 Xueyuan Road, Taiyuan, Shanxi 030051, China; ^2^Shanxi Province Cancer Hospital, 3 Zhigong New Street, Taiyuan, Shanxi 030013, China

## Abstract

**Objectives:**

To evaluate the utility of radiomics features in differentiating central lung cancers and atelectasis on contrast-enhanced computed tomography (CT) images. This study is retrospective.

**Materials and Methods:**

In this study, 36 patients with central pulmonary cancer and atelectasis between July 2013 and June 2018 were identified. A total of 1,653 2D and 2,327 3D radiomics features were extracted from segmented lung cancers and atelectasis on contrast-enhanced CT. The refined features were investigated for usefulness in classifying lung cancer and atelectasis according to the information gain, and 10 models were trained based on these features. The classification model is trained and tested at the region level and pixel level, respectively.

**Results:**

Among all the extracted features, 334 2D features and 1,507 3D features had an information gain (IG) greater than 0.1. The highest accuracy (AC) of the region classifiers was 0.9375. The best Dice score, Hausdorff distance, and voxel AC were 0.2076, 45.28, and 0.8675, respectively.

**Conclusions:**

Radiomics features derived from contrast-enhanced CT images can differentiate lung cancers and atelectasis at the regional and voxel levels.

## 1. Introduction

Central lung cancer is a type of cancer that may cause atelectasis, and atelectasis regions may be present around the tumor in central lung cancer [1]. Enhanced computed tomography (CT) imaging is a method recommended by NCCN for imaging examinations in patients with lung cancer [2]. In enhanced CT images, tumor regions and the atelectasis regions have a similar visual appearance; therefore, it is difficult to distinguish the two accurately, which can affect the delineation of the tumor boundary. Accurate delineation of the tumor boundary is of great significance in tumor diagnosis, staging, and treatment [3, 4].

Kovalev et al.'s study showed that statistical significance scores cannot effectively distinguish tumors from atelectasis regions on plain CT images, but methods such as generalized gradients can effectively enhance the distinction between tumor regions and atelectasis regions [5, 6]. Flechsig et al.'s study showed that the density analysis of plain CT images has a reference value for distinguishing tumors from atelectasis [7]. These findings prove the feasibility of distinguishing tumors and atelectasis on plain CT. Since the NCCN guidelines believe that enhanced CT is a stronger method of distinguishing tumors and atelectasis than plain CT, these studies also indirectly support the feasibility of distinguishing tumors and atelectasis on enhanced CT.

To study the distinguishability of tumors and atelectasis while avoiding the inefficiency and omissions of a manual feature analysis, we performed radiomics analysis of tumors and atelectasis on enhanced CT. Radiomics is a rapidly developing emerging field in medical imaging research and has great potential in analyzing medical images [8–12]. Radiomics has been proven to be an effective method in medical imaging research of the lungs and has been used in many applications [13–15]. Flechsig et al. explained the significance of density measurement in FDG PET/CT images for the N staging of lung cancer based on imaging omics methods [16]. Ahn et al. used imaging omics to predict the survival rate of patients after non-small-cell carcinoma tumor resection [17]. Li et al. explored the predictive ability of radiomics features based on 18F-FDG PET/CT images on the EGFR mutation status of non-small-cell lung cancer [18]. For diagnosis using clinical radiological imaging, there is often no manual delineation of suitable candidate regions, and only pixels (or voxels) are available for analysis. Therefore, studying the differentiation at the pixel level is of great significance in automated CT image analysis.

In this study, it is assumed that the features valid at the region level are still valid at the pixel level (or voxel level). Therefore, the region level is analyzed first, and then, the region-level method is transferred to the pixel level for verification. To measure the effectiveness of features and classification models, information gain (IG) [19–21] and machine learning methods are introduced.

In the clinical radiotherapy target delineation, the difficulty in distinguishing between atelectasis and tumor regions will lead to the need for patients to take multiple CT images. Even for some patients, nuclear magnetic image or positron emission tomography (PET) image other than CT image is necessary. The results of this research can be used as a reference for clinical radiotherapy target delineation and improve the delineation accuracy only based on single contrast-enhanced CT image. Therefore, the number of radiation exposures to patients can be reduced, and the diagnosis cost of patients can also be saved.

## 2. Materials and Methods

This retrospective study protocol was reviewed and approved by the institutional review board of our hospital. Written informed consent was waived.

### 2.1. Study Population

A total of 36 patients (4 females and 32 males; mean age 61.30 ± 7.66 years; range 43 to 73 years, as shown in Table 1) with central lung cancer and atelectasis between July 2013 and June 2018 were selected from the Shanxi Province Cancer Hospital.

The inclusion criteria were as follows: (1) diagnosis of central lung cancer, according to the standard diagnosis criteria [2]; (2) CT image showing atelectasis; (3) contrast-enhanced CT taken during the arterial phase; and (4) patients who were not receiving radiotherapy when the contrast-enhanced CT was obtained. Those with artifacts or poor image quality were not included in the study.

### 2.2. Image Acquisition

This section describes the scanning protocol.

Before scanning, we informed the patient and family members of the precautions during scanning and the risk of contrast injection. The scan will only be performed after the patient or family members have signed the informed consent form. Before the start of the scan, we will perform breathing exercises on the patient to reduce the influence of scanning motion artifacts. The patient took a supine position during the scan, with his hands raised above the top of his head, and was scanned from the entrance of the thorax to the bottom of the lung.

All contrast-enhanced chest CT images were acquired (on two GE Healthcare CT scanners) with the following parameters: 120 kV tube voltage, 300 mA effective power of tube, 1.375 pitch, 0.6 s/cycle rotation speed, 5 mm reconstruction slice thickness, 5 mm reconstruction slice interval, and 512 × 512 matrix. All images were scanned in a craniocaudal sense. Intravenous contrast media (1 mL/kg) was injected at a rate of 3.5 mL/s. The iodine contrast medium concentration used during CT scanning was 300 mg/mL. During the CT scanning, the bolus tracking was used, and the ROI was positioned on the descending aorta.

According to the position and size of the chest in the image, the field of view was uniformly set to 400 × 300.

### 2.3. Segmentation and Annotation

Two trained radiology physicians with more than 7 years of experience independently performed segmentation using the 3D Slicer (version 4.10.2, https://www.slicer.org/) [22]. The software interface of 3D Slicer is shown in Figure 1. The 3D Slicer can view DICOM format images and allows users to mark the images with voxel masks. The color patches on the enhanced CT image in Figure 1 are the results of the annotation. Difficult-to-identify lesions on contrast-enhanced CT were labeled with reference to the corresponding nuclear magnetic image or PET image. The identified tumor regions and the atelectasis regions were marked as masks separately. The region where the tumor and atelectasis are mixed was not specially marked but could be inferred from the confirmed tumor and atelectasis masks. Normal tissues and organs were not marked.

All masks are marked layer by layer and can be used directly in 2D analysis. The 3D masks are reconstructed from the 2D mask sequence. An example of data and masks is shown in Figure 2.

### 2.4. Radiomics Feature Extraction

The physicians performed segmentation mainly based on the 2D transverse plane of CT, but tumor regions and atelectasis regions are 3D objects. In cancer-related radiomics studies, the 3D shape features of a tumor are commonly used [23–26]. Kovalev et al.'s study explored the significance of 3D generalized gradient in tumor imaging research [6]. Guan et al.'s study showed that 3D radiomics features have certain reference values in distinguishing difficult-to-recognize boundaries [27]. To evaluate the effect of feature extraction in the two modes, features are extracted in 2D or 3D modes. In each mode, region-level feature extraction and pixel-level (or voxel-level) feature extraction were performed separately. When extracting voxel-level features from 3D images, since the ratio of the layer thickness to the pixel distance in the layer is not 1, the image data are resampled and corrected according to the actual ratio to prevent deviations in the radiomics analysis, therefore eliminating the anisotropy of the data format itself.

The extraction of radiomics features is divided into two steps: image transformation and feature calculation. The purpose of the image transformation step is to construct a feature map that is not linearly related to the original image. The feature calculation step calculates statistical features and texture features both on the original image and the transformed image. Extracting features from the transformed image essentially generates a large number of feature extractors through a nonlinear combination, which can make radiomics analysis more likely to obtain valuable features. The image transformation method used in this experiment is shown in Table 2, and the feature extraction methods used are shown in Table 3.

As some feature extraction operators cannot work with specific feature maps, the final number of features extracted is not equal to the product of the number of feature maps and feature extraction operators. Finally, 1,653 features were extracted based on 2D images and 2,327 features were extracted based on 3D images for analysis. The feature extraction program is based on Pyradiomics (version 3.0.1, https://pyradiomics.readthedocs.io/) [28].

To measure the significance of features in distinguishing tumors and atelectasis, the IG of each feature in the region classification problem was calculated using the following equations:

(1) $$\begin{array}{c} H\left(Y\right)=-\underset{y_{i}\in Y}{\sum }p\left(y_{i}\right)\log p\left(y_{i}\right),\\ H\left(Y\;|\;X\right)=-\underset{x_{j}\in X,y_{i}\in Y}{\sum }p\left(x_{j},y_{i}\right)\log\frac{p\left(x_{j},y_{i}\right)}{p\left(x_{j}\right)},\\ \text{IG}\left(Y\;\;|\;X\right)=H\left(Y\;\right)-H\left(Y\;\;|\;X\right), \end{array}$$

where *X* and *Y* represent random variables and IG(*Y* | *X*) represents the IG from *X* to *Y*. The greater the IG, the greater the effect of known *X* as a condition in determining *Y*.

Therefore, features with greater IG are considered to contribute more to classification. Theoretically, till the IG is nonzero, the features are related to the classification problem. To prevent errors caused by calculation and sampling from affecting the experimental results, in the classification problem (data distribution is uniform and the total entropy is close to 1), 0.1 is selected as the threshold (refer to the practice of Kim et al. [19]). Features with an IG less than 0.1 are considered irrelevant to classification.

### 2.5. Statistical Analysis and Machine Learning

Machine learning is a set of tools for understanding and modeling complex data [29]. Commonly used machine learning algorithms include random trees and random forests, support vector machines, and logistic regression. At present, various machine learning algorithms have been widely used in medical imaging-related research [30–36]. Machine learning algorithms are also often used as classifiers for radiomics research or as a means of evaluating radiomics analysis [37–39].

To verify whether the features selected according to the IG threshold are valuable for the classification of tumor regions and atelectasis regions, 10 machine learning models were trained based on features with an IG greater than 0.1. The indicators of these classifiers can illustrate the effectiveness of the selected features.

Pixel-level (or voxel-level) classifiers are trained on nonshape pixel-level (or voxel-level) features for further verification and to explore the feasibility of segmenting tumor regions from atelectasis regions. As each lesion region contains hundreds to thousands of pixels, the training cost of pixel classification is relatively large. For this reason, a commonly used data dimensionality reduction method, the principal component analysis algorithm (PCA), was adopted to reduce the dimension of data features and eliminate the correlation between data features. The main idea of PCA is to transform the data in the *n*-dimensional space into a new *k*-dimensional coordinate system. The *k* coordinate axes in the new coordinate system are the directions of the first *k* largest variance in the original data. When performing PCA, first, the *m* data is arranged into matrix *X* with *n* rows *m* column and the covariance matrix *C* is calculated using Equation (2). Then, the eigenvalues and eigenvectors of *C* are identified, and the eigenvectors are arranged into a matrix from top to bottom according to the size of the corresponding eigenvalues. Finally, the first *k* rows are taken to form a matrix *P* (generally select the eigenvalues with energy 99%), and the transformed data *Y* is calculated according to Equation (3).

(2) $$\begin{array}{c} C=\frac{1}{m}XX^{T}, \end{array}$$

(3) $$\begin{array}{c} Y=PX. \end{array}$$

To reduce the randomness of machine learning algorithms, all machine learning models have undergone fivefold cross-validation. Cross-validation is a method to verify the classifier, which can effectively reduce the false high phenomenon of the classifier index caused by model overfitting or accidental factors. That is, the data set is equally divided into five subsets, and five experiments are performed. Each time, a subset is selected as the test set, and the remaining subsets are combined as the train set for model training. After all experiments are completed, the results of five experiments are summarized to evaluate the model.

### 2.6. Model Validation

The indicators used to evaluate the pixel-level (or voxel-level) classifier are Hausdorff distance (HD), Dice score (DSC), and accuracy (AC). Suppose *X* is the real tumor region, *Y* is the tumor region predicted by the network, *d* represents the distance between two points, and *N* represents the number of pixels in the entire image. The calculation formula of HD is shown in Equation (4). The calculation formula of DSC is shown in Equation (5). The calculation formula of AC is shown in Equation (6).

(4) $$\begin{array}{c} \text{HD}\left(X,Y\right)=\max\left(\sup_{x\in X}\inf_{y\in Y}\;d\left(x,y\right),\sup_{y\in Y}\inf_{x\in X}\;d\left(x,y\right)\right), \end{array}$$

(5) $$\begin{array}{c} \text{DSC}\left(X,Y\right)=\frac{\left|X\cap Y\right|}{\left|X\right|+\left|Y\right|}, \end{array}$$

(6) $$\begin{array}{c} \text{AC}\left(X,Y\right)=\frac{\;|\;\left(X\cap Y\right)\cup \left(-X\cap -Y\right)\;|\;}{N}. \end{array}$$

## 3. Results

Lei et al.'s study explored the separability of tumors and atelectasis on contrast-enhanced ultrasound images [40]. There are similar studies on magnetic resonance imaging [41, 42]. Due to image differences, the results of these studies and ours are not comparable. Yang et al.'s study involves the distinction between tumors and atelectasis on CT images, but their study focuses on manual recognition and our research focuses on automatic detection [41]. Their study and ours are in different fields. Therefore, there is no comparability between Yang et al.'s study and ours. As far as we know, our study has no comparable study of its kind for now.

The data set of this study contains contrast-enhanced CT images of 36 patients with arterial stage central lung cancer. The patients included 4 females and 32 males. The age range of the patients is 43 to 73 years, and the average age is 61.30 ± 7.66. All contrast-enhanced chest CT images were acquired on two GE Healthcare CT scanners. Images with artifacts or poor quality were not included in this study.

### 3.1. Feature Information Gain

The distributions of the IG of features from 2D and 3D images are shown in Tables 4 and 5, respectively. To clarify the influence of the window level and window width on the experimental results in data preprocessing, a control experiment was carried out. CT images of the lungs are generally processed under the lung window. However, according to the experience of radiology physicians, a narrower window width can help distinguish tumors from atelectasis. Therefore, standard lung window (window width: 1,500 Hu, window level: -600 Hu) and empirical window (window width: 150 Hu, window level: 150 Hu) data were processed separately. In addition, data normalization is also used as an experimental variable to study the impact of data normalization on the results of radiomics analysis. Considering that the region shape features are important region features, but the shape features cannot be extracted at the pixel (or voxel) level, each experiment counts the total feature number and the number after removing the shape features.

Experimental results show that a large number of effective features (IG greater than 0.1) are extracted from both 2D and 3D data, but there are more effective features extracted from 3D data. Without normalization, it is easier to obtain valid data through the empirical window than the lung window. The impact of normalization on IG is more complicated. On the one hand, it will make the original data more regular, reduce abnormal and error values, and enlarge some feature differences. On the other hand, it also eliminates the physical meaning of the original data and causes the loss of some feature differences. Experimental results show that the effect of normalization on the empirical window is not as obvious as that of the lung window, which may be due to reducing the window width partly played a role in min–max normalization.

After weighing, the experience window data without normalization that can retain the physical meaning of the data were used for subsequent classifier training.

### 3.2. Building Region Classification Models

10 common machine learning models are trained on extracted features from 2D and 3D data (experience window, without normalization). In multiple comparative experiments, the IG threshold of the selected features was changed to study the influence of the IG threshold on the classification effect. The AC of the model under different conditions is shown in Table 6, and the maximum AC is 0.9305.

### 3.3. Building Voxel Classification Models

The effective features with IG higher than 0.1 are extracted at the voxel level (experience window, without normalization). These features are used to train the voxel classifier after principal component analysis. The experimental results of the voxel classifier are shown in Table 7.

## 4. Discussion

This retrospective study is a radiomics analysis of the tumor region and atelectasis region on the enhanced CT image. The results of this study can be used as references for the delineation of the radiotherapy target to improve the accuracy of target delineation based on enhanced CT. This will help reduce the patient's radiation exposure while saving treatment costs.

In the current literature that we know, there is no similar study that can be compared numerically with our study. At present, the study on the difference between atelectasis and tumor imaging features mainly focuses on the field of magnetic resonance imaging [41, 42]. There are few studies regarding the difference between tumor and atelectasis on enhanced CT images. Yang et al. explored the difference between tumors and atelectasis on CT images from the perspective of manual annotation [41]. Their study lacks an objective evaluation of imaging features, and our study objectively evaluated the differentiation effect of various imaging features on tumors and atelectasis through IG. In addition, we have also built machine learning models that can automatically classify tumors and atelectasis regions. Kovalev et al. demonstrated the value of generalized gradients for distinguishing tumors and atelectasis on CT images [5, 6]. However, their study only involves one image feature, while we tested thousands of features.

This study shows the following: whether it is 2D mode or 3D mode, a large number of effective features are extracted from contrast-enhanced CT images. The classifiers trained based on these effective features have reached a high AC rate, and the highest accuracy rate reached 0.9375. Since each patient has a tumor region and an atelectasis region, the ratio of the two regions is close to 1 : 1. Therefore, the region classification AC rate is considerably higher than 0.5, and a large number of effective features (measured by IG) can prove the differentiation of the tumor regions and the atelectasis regions on the contrast-enhanced CT image.

In the 3D mode, more effective features are extracted, and the classifier scores are higher. Therefore, the 3D mode is better than the 2D mode commonly used by radiology physicians when distinguishing tumors and atelectasis regions. As shown in Table 6, the score of some classifiers increases as the IG threshold increases. This could be because there are more significant associations that are easier to learn by machine learning models between features with higher IG and classification labels. Increasing the IG threshold enhances the effect of removing random factors to a certain extent.

After the experimental parameters obtained in the region analysis are transferred to the voxel level, sufficient effective features are obtained. The voxel classifier trained based on these features can achieve an AC rate of 0.8675. This proves the feasibility of using machine learning algorithms to segment tumors and atelectasis on contrast-enhanced CT.

The pathological types of central lung cancer are mostly small cell lung cancer and squamous cell carcinoma, and the same pathological type will have different degrees of differentiation. The main limitation of this experiment is that there is no distinction between pathological types. In the future, we will do further study on this.

The number of radiomics features tested in this study is very large but still cannot cover all possible features. Finding a more efficient feature test method to distinguish tumors from atelectasis is also the future direction of this study.

This study is based on enhanced CT images. Due to the change of CT value, when it comes to nonenhanced CT, the effective features on enhanced CT images do not necessarily remain effective. Due to the similar imaging methods, there is still a certain degree of similarity between contrast-enhanced CT and unenhanced CT [43–46]. Therefore, there is the possibility of migrating the effective features on enhanced CT to nonenhanced CT. However, the effect of migration needs to be verified by experiments.

## 5. Conclusions

This study analyzed the separability of lung tumor and atelectasis in contrast-enhanced CT, which directly facilitates CT diagnosis. Experimental data shows that tumors and atelectasis are separable at the region and pixel levels. It was found that tumors and atelectasis are easier to distinguish in 3D mode experience window (window width: 150 Hu, window level: 150 Hu) without data normalization.

A series of machine learning models that distinguish between tumors and atelectasis at the regional level and pixel level are constructed, establishing a theoretical foundation for artificial intelligence-assisted CT diagnosing and radiotherapy target delineation. This will help shorten the waiting time of patients, reduce unnecessary patient radiation exposure, reduce inspection costs, and improve the prognosis.

## Figures and Tables

**Figure 1:** 3D Slicer software interface.

**Figure 2:** An example of data and masks. (b, c, d) Red indicates tumor, green indicates atelectasis. (a) Original image. (b) Contours of tumor and atelectasis drawn by the physicians. (c) The masks generated from the contour. (d) 3D masks reconstructed from the 2D mask sequence.

**Table 1:** Population's characteristics.

Characteristics	Values
Mean age	61.30 ± 7.66
Age range	43 to 73
Sex ratio^∗^	4 : 32
Total patients	36

^∗^Indicates the ratio of women to men.

**Table 2:** Image transformation operations.

Transformation	Feature maps
Original	Original image
Wavelet	Wavelet decomposition subband^∗^
Log	Log processing results^∗∗^
Square	Square image
Square root	Square root image
Logarithm	Logarithm image
Exponential	Exponential image
Gradient	The gradient of the original image

^∗^Enhanced CT image data has 3 dimensions, and each dimension has two options of low-pass wavelet convolution and high-pass wavelet convolution, so there are 8 subbands in total. ^∗∗^Set the value of *σ* of the Log operator to 0.01, 0.1, 0.5, 1.0, 2.0, 3.0, and 5.0 to get 7 different processing results.

**Table 3:** Feature extraction operators.

Group	Feature extractor
Shape	VoxelVolume
	MeshVolume
	SurfaceArea
	SurfaceVolumeRatio
	Sphericity
	Max3DDiameter
	Max2DDiameterSlice
	Max2DDiameterColumn
	Max2DDiameterRow
	MajorAxisLength
	MinorAxisLength
	LeastAxisLength
	Elongation
	Flatness

Firstorder	Energy
	TotalEnergy
	Entropy
	Min
	10Percentile
	90Percentile
	Max
	Mean
	Median
	InterquartileRange
	Range
	MAD
	RobustMAD
	RootMeanSquared
	Skewness
	Kurtosis
	Variance
	Uniformity

GLCM	Autocorrelation
	JointAverage
	ClusterProminence
	ClusterShade
	ClusterTendency
	Contrast
	Correlation
	DifferenceAverage
	DifferenceEntropy
	DifferenceVariance
	JointEnergy
	JointEntropy
	Imc1
	Imc2
	Idm
	Idmn
	Id
	Idn
	InverseVariance
	MaxProbability
	MCC
	SumEntropy
	SumSquares

GLRLM	ShortRunE
	LongRunE
	GrayLevelNU
	GrayLevelNUN
	RunLengthNU
	RunLengthNUN
	RunPercentage
	GrayLevelVariance
	RunVariance
	RunEntropy
	LowGrayLevelRunEntropy
	HighGrayLevelRunEntropy
	ShortRunLowGrayLevelEntropy
	ShortRunHighGrayLevelEntropy
	LongRunLowGrayLevelEntropy
	LongRunHighGrayLevelEntropy

GLSZM	SmallAreaE
	LargeAreaE
	GrayLevelNU
	GrayLevelNUN
	SizeZoneNU
	SizeZoneNUN
	ZonePercentage
	GrayLevelVariance
	ZoneVariance
	ZoneEntropy
	LowGrayLevelZoneEntropy
	HighGrayLevelZoneEntropy
	SmallAreaLowGrayLevelEntropy
	SmallAreaHighGrayLevelEntropy
	LargeAreaLowGrayLevelEntropy
	LargeAreaHighGrayLevelEntropy

GLDM	SmallDE
	LargeDE
	GrayLevelNU
	DNU
	DNUN
	GrayLevelVariance
	DVariance
	DEntropy
	LowGrayLevelEntropy
	HighGrayLevelEntropy
	SmallDLowGrayLevelEntropy
	SmallDHighGrayLevelEntropy
	LargeDLowGrayLevelEntropy
	LargeDHighGrayLevelEntropy

NGTDM	Coarseness
	Contrast
	Busyness
	Complexity

**Table 4:** Feature number under different threshold of information gain on 2D images.

	With shape features				Without shape features			
	LW	LW, N	EW	EW, N	LW	LW, N	EW	EW, N
Total	1,653	1,653	1,653	1,653	1,638	1,638	1,638	1,638
0	1,564	1,193	1,483	1,317	1,551	1,180	1,470	1,304
0.1	139	170	344	170	134	165	339	165
0.2	4	4	14	4	0	0	10	0
0.3	0	0	0	0	0	0	0	0
0.4	0	0	0	0	0	0	0	0
0.5	0	0	0	0	0	0	0	0
0.6	0	0	0	0	0	0	0	0

LW: lung window; EW: experience window; N: normalized.

**Table 5:** Feature number under different threshold of information gain on 3D images.

	With shape features				Without shape features			
	LW	LW, N	EW	EW, N	LW	LW, N	EW	EW, N
Total	2,327	2,327	2,327	2,327	2,275	2,275	2,275	2,275
0	2,199	1,896	2,196	1,937	2,184	1,881	2,181	1,922
0.1	1,289	1,193	1,507	1,148	1,275	1,179	1,493	1,134
0.2	439	510	533	477	426	497	520	464
0.3	207	280	207	234	196	269	196	223
0.4	56	81	48	49	49	74	41	42
0.5	12	22	12	14	7	17	7	9
0.6	6	8	4	4	2	4	0	0

LW: lung window; EW: empirical window; N: normalized.

**Table 6:** The classification model accuracy result.

	2D			3D					
	0	0.1	0.2	0	0.1	0.2	0.3	0.4	0.5
Multilayer perceptron	0.3995	0.7493	0.6866	0.3458	0.3972	0.3319	0.3625	0.6694	0.6763
Decision tree	0.7352	0.7484	0.7045	0.8055	0.8472	0.7916	0.8333	0.8333	0.9166
Random forest	0.7845	0.7924	0.7361	0.8041	0.8375	0.8305	0.8527	0.8958	0.9111
AdaBoost	0.8122	0.7825	0.7132	0.8736	0.8708	0.8805	0.8805	0.8916	0.9375
Gradient boosting	0.7814	0.7831	0.71	0.8291	0.818	0.8333	0.8055	0.8319	0.8694
Bagging	0.7911	0.8143	0.7442	0.8375	0.8597	0.8486	0.8625	0.8708	0.8902
Bernoulli naive Bayes	0.6604	0.6603	0.3232	0.4166	0.5138	0.5694	0.125	0.8333	0.4583
Gaussian naive Bayes	0.7937	0.6942	0.7437	0.6805	0.6944	0.6805	0.6805	0.875	0.9305
Support vector machine	0.1129	0.1184	0.6628	0	0	0	0	0	0.1527
*K*-nearest neighbor	0.498	0.7209	0.6616	0.625	0.625	0.625	0.625	0.7222	0.8333

**Table 7:** The voxel classifier experiment results.

	DSC			HD			AC		
	Tumor	Atelectasis	Average	Tumor	Atelectasis	Average	Tumor	Atelectasis	Average
Decision tree	0.1886	0.2267	0.20765	78.6	40.63	59.615	0.8688	0.8217	0.84525
Random forest	0.1397	0.2244	0.18205	54.35	36.21	45.28	0.8988	0.8363	0.86755
*K*-nearest neighbor	0.1383	0.2059	0.1721	57.73	37.92	47.825	0.8875	0.8245	0.856
Gaussian naive Bayes	0.1305	0.1639	0.1472	63.08	40.23	51.655	0.727	0.6842	0.7056

## Data Availability

The raw/processed data required to reproduce these findings cannot be shared at this time as the data also forms part of an ongoing study.

## Abbreviations

CT: Computed tomography
AC: Accuracy
DSC: Dice score
HD: Hausdorff distance
IG: Information gain
NCCN: National Comprehensive Cancer Network.

## Additional Points

*Key Points*. Radiomics features are valuable in distinguishing atelectasis and central lung tumors on contrast-enhanced CT. Instead of manually selecting features one by one, we extract a large number of radiomics features and select effective features from them based on information gain. This method can cover as many feature types as possible and evaluate their values from the perspective of statistical information. Employing information gain and machine learning models, the accuracy rates of recognizing tumor regions and tumor region voxels reached 93.75% and 86.75%, respectively.
